# Measurement of the Correlation Degree between Rural Family Fertility Willingness and the Development of China's Labor Original Equipment Manufacturing Industry

**DOI:** 10.1155/2022/1062223

**Published:** 2022-05-26

**Authors:** Liangshan Li

**Affiliations:** Faculty of Public Administration, Shanxi University of Finance & Economic, Taiyuan 030006, Shanxi, China

## Abstract

At present, China is facing problems such as the decline of fertility rate, gender imbalance, serious aging, and the reduction of youth and working population, which will have an adverse impact on the long-term development of social economy. Based on the literature review, combined with China's financial family data, combined with the innovative calculation model of the correlation between rural family fertility willingness and labor original equipment manufacturing (OEM) industrial development, through the empirical analysis of rural families, this paper investigates the relationship between fertility willingness and the development and endogeneity of labor OEM industry and finds that female labor participation has a significant negative impact on the number of children in rural families. Spouse labor participation has a negative effect on the number of children in rural families. The regression coefficient of women's willingness to have two children for career development is significant and negative (*c*_1_=−0.181, *P*=−0.003 < 0.01), and that of women's family status is significant and negative (*c*_1_=−0.998, *P*=0.031 < 0.01). The relative opportunity cost of birth of individual operators is more concentrated in the range of 50%–80%. The results show that the development of labor OEM industry is significantly influenced by the fertility willingness of rural families. This paper concludes that differentiated policies and measures should be taken according to the type of industrial promotion.

## 1. Introduction

The introduction of the comprehensive three-child policy has greatly reformed the family planning policy that has been implemented for more than 30 years, which has attracted the attention of academia and the public. Some scholars worry that if the policy is liberalized, the pressure of fertility rate will still be great, and there will be another “population explosion.” Some scholars have high hopes for the two-child policy, which will significantly increase the fertility rate. The aging population will aggravate the decline of labor supply [1]. The working-age population is gradually decreasing, and the population distribution is gradually disappearing, as a result of the aging society. In this case, increasing the labor force participation rate of the working-age population, including women, is a key strategy for reversing the demographic dividend decline [2]. Population aging and disparities are becoming global concerns. Population decline and rapid aging result from a fertility rate below the replacement level. According to the World Bank database, the proportion of people under the age of 14 in the total population fell to 25.94 percent in 2017, while the proportion of people aged 65 and up rose to 8.70 percent [3, 4], indicating that the world is becoming an aging society. In this case, increasing the participation rate of the age-appropriate population, including women, in economic activities is an important way to offset the current decline in the demographic dividend, while increasing the fertility rate is an important way to offset future economic growth declines.

As the main body of reproductive behavior, women bear the dual roles of work and family, which is not only an important part of the labor market, but also an indispensable human resource for China's economic development and is responsible for the future labor supply and human resources. Fatima and others believe that the fertility rate depends on the balance between the income effect and the substitution effect of reproductive demand [5]. Devaro and others found that young women can delay or give up childbearing by learning the skills of reducing unemployment risk and increasing income [6]. Long believes that demographic dividend promotes economic growth by stimulating investment expansion, because it reduces the burden of dependence on the productive population and can spend more time and energy on productive activities, thus increasing investment and promoting the expansion of economic reproduction [7]. The research results of Mao et al. show that there is no direct relationship between female labor participation and fertility rate, and it is found that female labor participation has a positive impact on fertility rate [8]. The existing literature pays more attention to the relationship between female labor force participation and fertility rate in developed countries, but less attention to developing countries, especially China. China's fertility rate has been lower than the population replacement rate for many years, so there is concern about this phenomenon. Labor force participation rate and number of births: we do not pay attention to the comprehensive influence of women's labor participation on childbearing age and number of births.

Child support, fertility willingness, support, and other factors all play a role in the decision-making process for family fertility in rural areas. This paper adds to the explanation for the discrepancy between them, which is primarily due to women's reproductive choices in the labor market. The goal of this paper is to use the model in conjunction with data on female employment and fertility in China to better understand the impact of rural families' desire for children on the development of China's original equipment manufacturing industry, as well as to theoretically support the practical importance of family economic theory. Exploring how to eliminate the negative impact of women's employment on fertility through policy measures is useful for providing a theoretical foundation and decision-making reference for the government's employment policy direction and focus in the context of the current human dividend's disappearance.

Possible innovations of this paper are as follows:

1. A possible innovation of this paper is to link the influence of rural families' fertility willingness on the development of China's labor OEM industry with the demographic dividend, which is the growth source of the demographic dividend itself.
2. According to the research object, this paper adopts a variety of research methods, using probit and logit analysis methods as explanatory variables of children's binary variables, and the number of children is an ordinal variable analyzed by OLS. For different research objects, adopt more scientific analysis methods.

## 2. Related Work

### 2.1. Study on the Relationship between Fertility Willingness and Fertility Behavior

Fertility desire is people's desire and pursuit for fertility, and it is also the individual's desire and requirement for fertility, which is reflected in the expectation of the quantity, time, gender, and quality of fertility. Because there is a strong correlation between fertility behavior and fertility willingness, the three-dimensional thinking of fertility behavior is applied, in which fertility willingness, number of children, and gender of willing children are the main components.

In a high fertility environment, unexpected births often occur, and the actual number of children born is larger than the expected number. They think that the level of fertility willingness is much higher than the actual fertility rate. Yakita believes that the deviation degree of fertility will and behavior is influenced by the life cycle of women [9]. Tian et al. found that the implementation of the “two-child policy” gradually converged the willingness and fertility, and the proportion of “willingness is the same as action” and “willingness is less than action” gradually increased [10]. Erten and Metzger believe that men at the middle level of gender role equality are in the transitional stage from the traditional concept of gender role to the modern concept of gender role, facing a higher level of family and workplace conflicts [11]. This also means that both the concept of gender role equality and the traditional concept of gender role are helpful in increasing the fertility rate. Codazzi and others found that increasing women's labor force participation and educational opportunities would reduce women's willingness to have children, and at the same time strengthen women's position in rural families and give them more choices [12]. Shen et al. believe that unwanted fertility rate, gender preference, children's substitution effect and female age have significant influence on fertility rate [13]. Fin and others believe that the fertility rate will affect the employment of rural women, and the number of children will affect the working hours and income of rural women [14]. Rong and others believe that a family-friendly policy that only considers women's fair social status from the family perspective will have a negative impact on women's social status and further reduce the fertility rate [15].

### 2.2. Research on Labor OEM Industry

OEM industry, as its name implies, is an agent processing industry, also known as outsourcing industry, which is composed of many companies engaged in OEM industry. Its main business is to share the processing and assembly defects in other enterprises' industrial chains, and the main types are processing with incoming materials, processing with imported materials and processing with incoming samples. Labor cost is the main component of production cost. If the level of labor cost or labor wage rises, the production cost of enterprises will also rise. Industrial transfer is a process in which the market continuously allocates resources. Maximizing the allocation of resources through industrial transfer can promote the industrial structure of a country or region, improve efficiency, and ultimately promote economic development.

Harrison and others studied many companies and multinational corporations on the basis of empirical analysis and thought that, in the highly industrialized open economy, labor-intensive industries were easier to transfer than before [16]. Through historical and theoretical analysis, it can be seen that the industrial overlap formed by international industrial trade and international industrial investment is the basic condition of international industrial transfer, and international industrial transfer requires that the technical composition of goods produced be similar and different. In terms of the composition of values, Han et al. established a two-step game analysis framework and concluded that if the game was repeated twice, the refined Nash equilibrium result of the subgame of urban cooperation between the former industries could be obtained [17]. Yan and others suggested that local government transfer should not only consider regional economic interests, but also update ideas and build industrial parks on the basis of cooperation to achieve win-win results [18]. Huang pointed out that enterprises may “escape” from the investment competition among local governments and emphatically analyzed the dynamic game process between local governments and enterprises and between local governments in the investment competition [19].

## 3. Methodology

### 3.1. Model Design

Analyzing the factors affecting fertility will help systematically understand the three child policy support needs of people of childbearing age. Through the analysis of the “three-child” policy and the wishes of children of childbearing age groups, it can be seen that the “three-child” policy is an important measure to solve the problems of China's population structure and population aging. The three-child policy is facing the dilemma of low fertility willingness, which is not conducive to the healthy development of China's society and economy [20].

I can divide the influencing factors into the following:

1. The main economic factors are high economic pressure and high cost of raising three children.
2. Social factors, including raising children to prevent old age, giving birth to elders, happy and complete family, unattended children, affecting the development of work and career, etc.
3. Cultural factors, such as the hope of both children and children to satisfy parent-child feelings.

Due to the needs of China's actual national conditions, the family planning policy is China's basic national policy, and the influence of policy factors on fertility willingness of fertility families is also worth investigating. Therefore, this study divides the influencing factors of childbearing families into four dimensions: policy factors, economic factors, social factorsm and cultural factors. The theoretical framework of this paper is shown in Figure 1.

In order to observe the influence of rural families' fertility desire on the development of China's labor OEM industry, it is assumed that women decide both the employment situation and the childbearing time and that she has not changed her employment situation after giving birth to her first child, and she decides whether to work at the same time as giving birth to her child. Assume that the number of children and women employed in a given period is the result of this decision-making process.

The independent variable is the number of children in rural families, represented by *Y*_th_, *t* is the time variable, and *h* is the family variable. The expectation of *Y*_th_ based on the exogenous feature *z*_th_ is represented by *E*[*Y*_th_*|Z*_th_, *θ*] and *θ*. According to the above model and iterative expectation law, the conditional expectation of *Y*_th_ can be obtained as follows:

(1) $$\begin{array}{c} E\left[Y_{th}|Z_{th},\theta \right]=E_{I_{\left(Y_{th}>0\right)},W_{th}}\left[E\left[Y_{th}|I_{\left(Y_{th}>0\right)},W_{th},Z_{th};\theta \right]|Z_{th};\theta \right], \end{array}$$

*W*_*th*_ represents the situation of women's employment (*W*_*th*_=1 means women's employment, 0 means other). *I*_(*Y*_*th*_ > 0)_ is the index function of children's existence.

Basically, the fact that the unobservable factors that determine women's employment status have nothing to do with whether they have children or not is not included in this model. Different from the case of univariate (probability and logarithm), the comparison between bivariate linear and multinomial logarithmic models is complicated, and there is no direct connection between the parameter estimates obtained from the two models. When children enter rural families, their conditional expectations are

(2) $$\begin{array}{c} E\left(Y_{\text{th}}|W_{\text{th}}=1,I_{\left(Y_{\text{th}}>0\right)}=1;Z_{\text{th}},\beta_{1}\right)=1-\exp\left(Z_{\text{th}}^{'}\beta_{1}\right). \end{array}$$

For the existence of the second child, this setting always has an expected value greater than 1, which is limited by the existence of the child.

First, we examine the variables related to the number of children in rural families. The variable described in this paper is the fertility rate, which is a binary dummy variable with a value of 1 when a child is born. The model of logit, probit regression, is

(3) $$\begin{array}{c} Y_{th}=\alpha_{0}+\alpha_{1}{\text{jobstatus}}_{h}+\alpha_{2}{\text{fjobstatus}}_{h}+\alpha_{3}{\text{fincome}}_{h}+\alpha_{4}{\text{wage}}_{h}+\alpha_{5}{\text{family}}_{h}+\mu_{h}. \end{array}$$

The variables in the model are explained in Table 1:

There is a causal relationship between rural family fertility willingness and the development of Chinese labor OEM industry. The choice of female reproductive behavior mainly includes the choice of reproductive age and the choice of the number of children, which is also a process of mutual decision and influence. Based on this, this paper constructs the following simultaneous equations to evaluate the influence of women's labor participation behavior on the childbearing age and the number of children.

(4) $$\begin{array}{c} {\text{Number}}_{\text{it}}=\alpha_{0}+\alpha_{1}{\text{Labor}}_{\text{it}}+\alpha_{2}{\text{Age}}_{\text{it}}+\alpha_{3}X_{\text{it}}+\alpha_{4}U_{\text{it}}+\alpha_{5}P_{\text{it}}+\mu_{\text{it}},\\ {\text{Age}}_{\text{it}}=\beta_{0}+\beta_{1}{\text{Labor}}_{\text{it}}+\beta_{2}{\text{Number}}_{\text{it}}+\beta_{3}Y_{\text{it}}+\beta_{4}U_{\text{it}}+\mu_{\text{it}}\text{.} \end{array}$$

Among them:

 
Number_it_,Age_it_—Representing the number and age of women's childbearing respectively is the main index of reproductive behavior choice.
 
Labor_it_—Variables reflecting women's labor participation, in this study, we will mainly consider whether women participate in labor and the nature of labor as variable indicators.
 
*X*_it_—Personal characteristics affecting the number of births.
 
*Y*_it_—Personal characteristics that affect the reproductive age.
 
*U*_it_—Other controlled variables, mainly including the characteristics of family and community.
 
*P*_it_—Virtual variable of family planning policy.

It can provide nonagricultural employment opportunities for surrounding women as a leader in economic development, and because of its proximity, it can also promote rural women's participation in nonagricultural work, which is beneficial to local rural women's participation in nonagricultural work. It is a problem that women should not consider when making reproductive decisions, just as it is a problem that women should not consider when making transportation facilities such as bus stops, development zones, and special economic zones. It only has to do with labor participation in decision-making and has nothing to do with reproductive choices.

We constructed a dynamic two-person and three-level game with complete information [21]. The competing government *A* and the company are located in the middle, and the company has three optional operations: requirement and default, *A*. The government adopts two selective measures to increase the preferential margin and maintain the status quo.

If the enterprise fails to ask government *A* to provide more preferential treatment, otherwise, it will move to Zhengzhou. Government *A* learns that government *B* has also implemented preferential policies for attracting investment. At this time, the economic aggregate of the enterprise is (*R*+*E*_3_), the economic aggregate of government *A* changes to (*G*_1_ − *E*_3_), and the economic aggregate of government *A* does not change to *G*_2_, with zero change.

In the third stage, the enterprise's strategies are migration, default, and requirements. At the time of migration, the economic aggregate of enterprises is (*R*+*E*_2_ − *C*), the economic aggregate of government *A* is (*G*_1_ − *R*), and that of government *B* is (*G*_2_+*R* − *E*_2_).

If the enterprise chooses the default at this time, the economic aggregate of the enterprise is (*R*+*E*_1_), the economic aggregate of government *A* is (*G*_1_ − *E*_1_) at this time, and the economic aggregate of government *B* remains unchanged. This cycle continues until a certain local government withdraws from the game process. The whole game process is shown in Figure 2:

*A* ^0^ is defined as the game in which government *A* starts bidding. Because the whole game process is repeated indefinitely, *A*^0^ does not affect the game analysis process at any stage. In this game, enterprises can freely choose whether to suspend negotiations with government *A* and turn to other regional governments.

Let *π*^0^ be the upper bound of the payment that enterprises can get in this game equilibrium. We use *A* to represent the game that the enterprise has stopped the negotiation and turned to government *B* to renegotiate, and also let *π* represent the upper bound of the payment that the enterprise can get in equilibrium. We can clearly show the process of the stage game we intercepted with Figure 3 below.

In this model, we also need the following two constraints:

After bidding, the enterprise must wait for the counteroffer of government *A*, which is in the position of “insider,” before deciding whether to suspend negotiations with it and start negotiations again with new “insider.” The negotiation between an enterprise and a certain government must last at least *T* time periods.

In game *A*^0^, enterprises choose their own payment maximization, so there are

(5) $$\begin{array}{c} \pi^{0}=\max\left(\sigma_{1}\left(1-\sigma_{2}+\sigma_{2}\pi^{0},\pi \right)\right). \end{array}$$

Because *π* is the supremum of the solution in game *A* equilibrium, so

(6) $$\begin{array}{c} \pi =\frac{\left(1-\sigma_{2}\right)\left[1-{\left(\sigma_{1}\sigma_{2}\right)}^{T+1/2}\right]}{1-\sigma_{1}\sigma_{2}}+\sigma_{1}^{T-1/2}\sigma_{2}^{T+1/2}\pi^{0}. \end{array}$$

According to (5), if *π*^0^=*σ*_1_(1 − *σ*_2_+*σ*_2_*π*^0^), there is

(7) $$\begin{array}{c} \pi^{0}=\frac{\sigma_{1}\left(1-\sigma_{2}\right)}{1-\sigma_{1}\sigma_{2}}. \end{array}$$

Substituting (7) into (6) results in

(8) $$\begin{array}{c} \pi =\frac{1-\sigma_{2}}{1-\sigma_{1}\sigma_{2}}. \end{array}$$

If *π*^0^=*π* is substituted into formula (6), the maximum payment of the enterprise is

(9) $$\begin{array}{c} \pi =\frac{\left(1-\sigma_{2}\right)\left[1-{\left(\sigma_{1}\sigma_{2}\right)}^{T+1/2}\right]}{\left[1-\sigma_{1}\sigma_{2}\right]\left[1-\sigma_{2}{\left(\sigma_{1}\sigma_{2}\right)}^{T-1/2}\right]}. \end{array}$$

At this time, the payment of government *A* is 1 − *π*.

Through the analysis in the last part, we compare the labor cost, land cost, and tax preference of the two places to illustrate the main differences of the expected profits of enterprises in the two places.

Random forest (RF) algorithm is an ensemble learning algorithm based on decision tree. Decision tree is a single learning method, called “Basic Learner,” which combines multiple decision trees into a “Forest.” By forming a strong learner in the integrated learning method, the predictive ability of the algorithm can be effectively improved. Create RF model:

(10) $$\begin{array}{c} y_{n}=f^{*}\left(\cdot \right)=\sum_{b=1}^{B}f^{b}\frac{\left(n,x,x_{i},t_{i},T,\lambda \right)}{B}. \end{array}$$

Among them, *x*_*i*_, *t*_*i*_ are the characteristic variable and the corresponding splitting critical value of each decision tree when splitting at the *i*-layer in RF algorithm according to the principle of “minimizing the sum of squares of residuals.”

 
*λ*—The punishment intensity of complexity *T* obtained by cross-validation method;
 
*n*—Core characteristic variables;
 
*x*—Other characteristic variables;
 
*B*—Number of decision trees contained in RF.

After obtaining the results of parameters such as *x*_*i*_, *t*_*i*_, *T*, *λ* through algorithm training and verification, the relative opportunity cost of childbearing can be combined with the level of living burden to measure the degree that the opportunity cost of childbearing can be borne.

### 3.2. Data Source and Variable Description

The data used in this paper is the panel data of CFPS 2015–2021. In this study, the variables used in the equivalence scale method include income satisfaction, total family income, family size, and number of children. This paper chooses income satisfaction as the explanatory variable. We need to filter data and delete missing items and outliers of families with children under 20 years old. Because the answer of income satisfaction is set to 1 to 5, 1 means “unsatisfied,” and 5 means “very satisfied,” and the variable is discrete.

Compared with cross-sectional data, panel data has certain advantages: first, it can use the difference between groups to multiply the time trend, so as to eliminate the possible deviation caused by small samples; secondly, the endogenous problem can be overcome by using lag data.  Table 2 reports the descriptive statistics of the main variables.

Among the basic elements of social support, this paper takes into account the respondents' maternity insurance status, peer reproductive pressure, and local infant community service facilities.  Table 3 shows descriptive statistics of independent variables of basic state characteristics of social support.

From Table 1, we can see that most people still choose to enjoy maternity insurance, which may be because many people in this survey are in economically developed areas, and maternity protection in these provinces and cities is in place. According to Table 2, it is found that many respondents have fertility pressure. When processing the data, the author assigns the answers of “absolute influence,” “greater influence,” and “general” as 1. Infant service facilities have a great influence on fertility willingness, otherwise, 2. Infant service facilities have little influence on fertility willingness.

## 4. Experiment and Results

Increasing the female labor force participation rate can revitalize the current economy, but it will significantly reduce the female fertility rate, further affect the national fertility rate, and affect the future labor supply and economic development. Therefore, it is the goal of all countries to maintain a high female labor force participation rate without affecting the fertility rate. Asian countries, especially some East Asian countries and Southeast Asian countries, should constantly improve policies to encourage women to bear children, such as parental leave and flexible working system.

The regression results in Figure 4 show that women's career development has a significant negative impact on the fertility willingness of the two children, and the rise of women's family status plays a part of the intermediary role.

The regression coefficient between women's career development and their willingness to have two children is significant and negative (*c*_1_=−0.181, *P*=−0.003 < 0.01), indicating that the better the career development, the lower the probability that women intend to have two children. The regression coefficient between women's family status and the willingness to have two children is significant and negative (*c*_1_=−0.998, *P*=0.031 < 0.01), indicating that the higher the family status, the lower the probability that women intend to have two children. This means that the impact of a woman's professional advancement on her desire to have two children is at least partially realized through the parameters of her family status. The improvement of women's family status is one of the negative effects of their career advancement on their willingness to have a second child. We made a comparison by age in Figure 5 to explain in detail the fertility wishes, current fertility behaviors, and future fertility plans of these women.

The following points can be observed from Figure 5:

1. There are differences in women's fertility wishes of all ages, but the differences are not too great, fluctuating around 1.5.
2. Compared with women in other age groups, the 20–24 age group has the lowest willing fertility rate.
3. The gap between the maximum and minimum target fertility rate of women gradually narrows with the increase of age, which indicates that the younger the women, the greater the variability of family planning.
4. With the increase of age and the distance between women's fertility ideal and future fertility plan, the possibility of realizing fertility ideal also increases. Women of different ages were born in different ages, and their fertility wishes, current fertility behaviors, and future fertility plans all reflect the differences among women of different ages.

From the calculation results of social support status factor model, it can be seen that the social support factors selected in this study have no significant influence on the fertility desire of childbearing age families. The coefficient of maternity insurance coefficient is negative, and respondents without maternity insurance are more likely to have children, which may be because people without maternity insurance are often distributed in rural areas.

Age can have relatively traditional thinking. In addition, the above results can be obtained because the coverage rate and wages of maternity insurance are generally low, which can not be used as the guarantee of fertility (Figure 6).

Peer pressure factors have no significant influence on the willingness of families to bear children, and the absolute value of the coefficient is very small, which is 0.009, which may be the reason for sample selection. In addition, as shown above, it is found that the factors of infant service facilities in local communities have no significant influence on the family's fertility desire, which may be due to the imperfect infant service facilities in China. Many families of childbearing age with better economic conditions look for private kindergartens and other childcare facilities at their own expense, while families with poorer economic conditions often choose families. Therefore, for families of childbearing age, the factors of infant service facilities in local communities are very important, and the fertility will has no significant influence.

The difference of reproductive opportunity cost of women in different education levels and employment units also confirms the role of maternity insurance. As shown in Figure 7, on average, women with lower education level have higher absolute and relative opportunity cost of childbirth.

Women with master's and doctor's degrees have the lowest absolute and relative opportunity cost of childbirth, and this group of women is more likely to engage in high-paying jobs with high working threshold and high maternity insurance coverage. Because of the high opportunity cost of fertility rate, social security is not perfect.

Figure 8 shows the reproduction opportunity cost of employers according to the nature of legal entities. Figures 8(a) and 8(b) show that the relative opportunity cost of female fertility rate in public units is more obviously concentrated in the range of 0–10%, while that in private units is concentrated in the range of 10%–20%. The relative opportunity cost of female fertility rate of local governments and social organizations is concentrated in the range of 0∼10%, which is distributed symmetrically around 0. However, the relative opportunity cost of female fertility rate of self-employed households is concentrated in the range of 50%∼80%. Compared with other types of units, self-employed households cannot protect their own rights and interests because they do not buy maternity insurance.

According to the regression results, female labor participation has a significant negative impact on the fertility level of one and two children. In the regression process, the regression results obtained by probit and logit are consistent. In order to ensure the reliability of regression results, this paper uses OLS to test the robustness of probit regression results. The obtained test results are shown in Table 4, and the obtained results are remarkably consistent, and the regression results are stable.

Combined with the research direction of this paper and the availability of selected data, this paper chooses the number of elderly people in rural families as the tool variable of female labor supply model. The results are shown in Table 5.

The endogenous relationship between women's labor participation rate and fertility rate is solved using the instrumental variable method, and the rural elderly population is used as an instrumental variable in regression estimation. Female labor participation has a significant negative impact on one or two child fertility rates. The negative impact of women's labor on the two children is particularly significant in the empirical findings. An important reference is how to improve the three-child fertility rate in the context of China's three-child policy liberalization.

## 5. Conclusions

The research of this paper mainly focuses on the measurement of the correlation degree between rural families' fertility willingness and the development of China's labor OEM industry and investigates the main influencing factors of different children in rural families. The main findings are as follows:

1. The regression analysis results considering the influence of female labor participation on fertility rate show that female labor participation has a significant negative effect on the number of children in rural families, and female labor participation will lead to the decrease of the number of children in rural families.
2. The regression coefficient between women's career development and their willingness to have two children is significant and negative (*c*_1_=−0.181, *P*=−0.003 < 0.01), indicating that the better the career development, the lower the probability that women intend to have two children. The regression coefficient between women's family status and the willingness to have two children is significant and negative (*c*_1_=−0.998, *P*=0.031 < 0.01), indicating that the higher the family status, the lower the probability that women intend to have two children.
3. The relative opportunity cost of unit female fertility rate is more obviously concentrated in the range of 0–10%, while that of private ownership is concentrated in the range of 10%–20%. The relative opportunity cost of female fertility rate in local governments and social organizations is concentrated in the range of 0∼10%, and distributed symmetrically around 0, but the relative opportunity cost of self-employed fertility rate is in the range of 50%–80%.

## Figures and Tables

**Figure 1:** An analysis framework of influencing factors of childbearing family's fertility willingness.

**Figure 2:** The second stage game process.

**Figure 3:** The process of intercepting stage game.

**Figure 4:** The influence of women's career development and family status on the fertility willingness of two children.

**Figure 5:** Women's will, current and target age-specific fertility rate in line with the two-child policy.

**Figure 6:** Social support condition factor model.

**Figure 7:** Differences in reproductive opportunity cost of women with different educational levels.

**Figure 8:** Comparison of reproductive opportunity cost of women in different employment units.

**Table 1:** The variables in the model.

Variable	Explaining variables
*Y*_th_	The number of children in rural families, *h* is the family variable
jobstatus	Female labor participation
fjobstatus_*h*_	Employment of fathers in rural families
fincome_*h*_	Per capita household income of the sample
wage_*h*_	Binary explanatory variable
family_*h*_	Other influencing factors in rural families that affect fertility rate
*μ*_*h*_	The number of children in rural families is an orderly variable.

**Table 2:** Descriptive statistics of main variables.

Variable	Mean value	Standard deviation	Observation and measurement
Total fertility rate *T*	3.15	1.32	1136
Female labor participation rate *F*	44.1	20.01	1427
Proportion of urban population to total population *C*	50.31	25.68	1427
Neonatal mortality rate *B*	33.21	27.14	1427
Female primary school enrollment rate *S*1	95.32	20.63	1021
Female secondary school enrollment rate *S*2	72.4	26.74	886
Enrolment rate of female colleges and universities *S*3	22.17	17.16	653

**Table 3:** Support independent variable description statistics of basic social situation characteristics.

Independent variable	Variable assignment	Minimal	Maximum	Mean value	Standard deviation
Is there maternity insurance *Q*	1 = yes	1	2	1.33	0.412
	2 = No				

Peer fertility pressure *W*	1 = yes	1	2	1.06	0.364
	2 = No				

Influence of infant service facility on fertility willingness *E*	1 = greater impact	1	2	1.27	0.428
	2 = minor impact				

**Table 4:** Influence of labor supply on fertility level.

Variable	A family with one child	Families with a second child
*T*	−0.06^*∗∗∗*^	−0.097^*∗∗∗*^
*F*	0.121	0.041^*∗∗∗*^
*C*	−0.002^*∗∗∗*^	−0.066
*B*	−0.006	−0.001^*∗*^
S1	0.017	−0.017
S2	−0.009	0.068
S3	−0.047	−0.087^*∗∗∗*^
*Q*	−0.367^*∗∗∗*^	−0.201
*W*	0.001^*∗*^	−0.002^*∗∗∗*^
*E*	−0.038	−0.047

Note: ^*∗*^, ^*∗∗*^ and ^*∗∗∗*^ are significant at the level of 10%, 5% and 1% respectively.

**Table 5:** Influence of labor supply on fertility level.

Variable	A family with one child	Families with a second child
Number of elderly people in rural families	2.318^*∗∗∗*^	2.217^*∗∗∗*^
Labor supply	−0.036	−0.863^*∗∗∗*^
Average personal household income	−0.128	−0.221
Is there any wage income	−0.001	−0.003^*∗*^
Total cash and deposits	−0.068^*∗∗*^	−0.012^*∗∗∗*^
Account status	−0.042	−0.076
Age	−0.033^*∗∗∗*^	−0.038^*∗∗*^
Gender	0.168	−0.156

## Data Availability

The data used to support the findings of this study are available from the corresponding author upon request.
